# Composition, Biogenesis, and Role of Exosomes in Tumor Development

**DOI:** 10.1155/2022/8392509

**Published:** 2022-09-09

**Authors:** Leila Moeinzadeh, Iman Razeghian-Jahromi, Zeinab Zarei-Behjani, Zohreh Bagheri, Mahboobeh Razmkhah

**Affiliations:** ^1^Department of Tissue Engineering and Applied Cell Sciences, School of Advanced Medical Sciences and Technologies, Shiraz University of Medical Sciences, Shiraz, Iran; ^2^Shiraz Institute for Cancer Research, School of Medicine, Shiraz University of Medical Sciences, Shiraz, Iran; ^3^Cardiovascular Research Center, Shiraz University of Medical Sciences, Shiraz, Iran

## Abstract

The role of exosomes and their mechanism of action at the tumor site have received increasing attention. These microvesicles are produced by a wide range of cells including mesenchymal stem cells (MSCs) and immune cells. In particular, tumor cells release remarkable amounts of exosomes which spread to distant organs through the blood and enhance the possibility of tumor metastasis. In spite of results on tumor promoting properties, there are reports demonstrating the tumor inhibiting effects of exosomes depending on the type of the tumor and cell source. This review aims to have a comprehensive appraisal on the biogenesis, composition, and isolation of exosomes and then highlights the current knowledge of their role in cancer progression or inhibition by special focusing on MSC's exosomes (MSC-EXOs).

## 1. Background

Paracrine factors like exosomes, which are produced by various types of cells such as mesenchymal stem cells (MSCs), immune cells, and tumor cells in the tumor microenvironment (TME), are emerging as a new communication system between cells involved in supporting tumor progression through the production of several cytokines, chemokines, and growth factors [1]. Cross-talk between cells of TME such as MSCs and tumor cells also seems to be pivotal for tumor growth and expansion. In 2010, MSC-EXO was firstly described in a mouse model of myocardial ischemia/reperfusion injury [2]. Relevant studies in this field represent that MSCs transmit signal molecules that regulate proliferation, angiogenesis, and metastasis of tumor cells by producing exosomes and controlling many cellular pathways. Now, whether exosomes from different sources strengthen or inhibit tumors is debatable, and many studies have reported unpredictable conclusions [3, 4]. This review presents the classification, preparation and characterization, storage stability, and biomarkers of exosomes and also emphasizes on the current evidence about MSC-derived exosomes in cancer progression.

## 2. Main Text

### 2.1. Extracellular Vesicles (EVs)

In 1967, Wolf firstly investigated platelet-derived vesicles with coagulant properties. In 1970s, EVs were described as a group of cell-derived structures [5], and extra roles of EVs were regularly discovered in the next years [6]. Now, EVs are usually viewed as significant mediators of cell signaling, but because of their remarkable heterogeneity, the mechanisms of this signaling pattern is unclear [7, 8]. In 2011, the International Society for Extracellular Vesicles (ISEV) recommended “Extracellular Vesicle” (EV) as the universal term for all membrane vesicles that are secreted into the cell environment [9, 10]. Despite the lack of diagnostic tools, recent evidence showed that EVs' subpopulations differ in biophysical features, proteomic content, and RNA receptors. EVs oscillate from 30 to 1,000 nm in size. Kowal and colleagues suggested that there are three sizes of EVs (large, medium, and small) which can be isolated by low, intermediate, and high-speed centrifugation, respectively. Among the small-EVs, four subcategories were defined by their degree of CD63, CD9, and/or CD81 tetraspanin expression [11, 12]. Recently, interest in EVs research has increased exponentially, and more efforts have been made to accurately understand the performance of EVs [9, 10]. They have been shown to be associated with various cells in the body as a new mechanism of intercellular communication and are presently accepted as the sources of circulating disease biomarkers [13–15]. Extracellular vesicles are extremely conserved in both eukaryotes and prokaryotes and released by many cell types, and both normal and dying cells discharge membrane-bound vesicles. EVs can cause various effects, protective, and pathologic, depending on the specific condition [16]. EVs are mostly allocated into three subgroups depending on their size, biogenesis, and deposited cargo composition [17]: (a) exosomes, 40–150 nm, which create from the inside budding of the late endosomal membrane, (b) ectosomes or microvesicles, 150–1000 nm, generating from direct budding of the plasma membrane and finally, (c) apoptotic bodies that have a broad size, 100–2000 nm, and released from apoptotic cells [15, 18]. Extravesicle subtype characteristics are shown in Table 1. Among EVs, exosomes have received particular attention in recent decades [19, 20].

### 2.2. History of Exosomes

Exosomes were first observed in the early 1980s [33]. In 1981, Trams et al. generally introduced exosomes as plasma membrane-derived vesicles with 5′-nucleotide enzyme activity with physiological functions [34]. Exosomes with conserved structures formed in the diverse of cells, they were identified over 25 years ago through the development of erythrocytes [35].

Johnston et al. traced receptors of transferrin during reticulocyte maturation and found that exosome formation was lost by transferrin receptors-mechanism in mature red blood cell process. The transferrin receptor, as one of the proteins on the surface of reticulocytes, disappears from the reticulocyte membrane upon red blood cells maturation. Selective loss of membrane proteins occurs with the formation of multicellular bodies (MVBs). Also, in the blood, which contains reticulocytes, circulating vesicles (exosomes) that contain specific proteins such as transferrin receptors and lipids of the plasma membrane are clearly seen [36]. Based on ISEV 2018 guidelines, the term “exosome,” in spite of widespread use, has been replaced by “small extracellular vesicles (sEV)” [37]. However, they have emerged as intercellular courier orchestrating a variety of cellular processes which might affect both neighboring environment and distant parts of the body [38, 39]. The size of exosomes is measured about 40–150 nm and fluctuates with a density gradient of sucrose at a density of 1.13–1.19 g/ml, and their morphology was reported as typical “cup-shaped” [40]. They are categorized into nine groups based on the morphology, single vesicle, double vesicle, triple vesicle or more, small double vesicle, oval vesicle, small tubule, large tubule, incomplete vesicle, and pleomorphic vesicle [41, 42].

Exosomes can actively be produced under normal or pathological conditions from different types of cells such as human umbilical vein endothelial cells, reticulocytes, and immune cells such as T and B lymphocytes, macrophages, dendritic cells (DCs), natural killer (NK) cells [43, 44], stem cells, fibroblasts, endothelial cells, epithelial cells, and neuronal cells [2, 45]. They are enriched with biologically active substances and can act as biological messengers for intra- and intercellular communication. By transferring biomolecules from parental cells to recipient cells, exosomes can play a fundamental role in tumor biology [23].

### 2.3. Exosome Biogenesis, Release, and Uptake

Due to their small size, exosomes easily escape from macrophage-dependent phagocytosis and pass easily through the walls of blood vessels and extracellular matrix. Surface expression levels of CD55 and CD59 help them to avoid activation of opsonin and coagulation factors. Accordingly, they can be broadly dispersed and stabilized in biological fluids. In fact, the existence of various proteins on their surfaces simplifies entering to the cells in a range of mechanisms after binding the cells. One of the main ways of exchanging information between exosomes and target tissues is receptor-mediated endocytosis, which effectively leads to a continuous and stable transfer of contents into the blood. In addition, exosomes with a high ability to target tissues or cells can easily cross biological barriers such as the blood-brain barrier; thus, make it possible to use them as hopeful drugs for transferring biomaterials in different situations [44, 46].

The exosome development contains four phases as follows: initiation, endocytosis, multivesicular body development, and release. The formation of exosomes begins with endocytic vesicles through invagination of the cell membrane toward forming early sorting endosomes (ESEs) that later develop into late sorting endosomes (LSEs) [4]. LSEs then undergo inward budding leading to the formation of multivesicular bodies (MVBs) which then fuse with the plasma membrane and release their contents into the extracellular environment which are now called exosomes. Next, released exosomes are directed to other cells possibly through some cell surface proteins such as tetraspanins [13, 47, 48] (Figure 1).

In this way, MVBs are generated through two mechanisms [49] including endosomal sorting complexes required for transport dependent (ESCRT) and ESCRT-independent mechanisms. The ESCRT dependent pathway is activated by a set of cytoplasmic protein complexes (ESCRT-0, ESCRT-I, ESCRT-II, and ESCRT-III) that identify ubiquitin-modified membrane proteins. They are required for exosome biogenesis [50]. In ESCRT-independent mechanism, the alg-2 interacting protein X binds to adaptor proteins inside the cell and contributes to the formation of exosomes. Production of these ESCRT-independent MVBs induces MVB formation through tetraspanins and ceramide-induced cell membrane germination [4]. There are reports introducing specific structures such as four-transmembrane domain proteins and lipid raft which have important roles in the formation of some exosomes [44, 49, 51]. Exosomes transmit information to the recipient cells through three main pathways: (1) receptor-ligand interaction, (2) straight merging with cell membrane, and (3) endocytosis via phagocytosis. Also, there are several proteins that act as specific receptors to activate the uptake of the exosome, such as ICAM-1 for antigen-presenting cells (APCs) and Tim 1/4 for B-cells [52].

### 2.4. Methods for Characterization, Isolation, and Analysis of Exosomes

Features of exosomes are correlated with their cell origin. Totally, the MSC-EXOs express CD63, CD9, and CD81 markers; however, the human umbilical cord-EXOs specially express Hsp70 and TSG101 proteins as well as some adhesion molecules including CD29, CD44, and CD73 [20, 53, 54]. The MSC-EXOs exhibit round morphology with the average size of 48.72 ± 2.7 nm. The major peak in particle size was assumed at 65–75 nm, and the overall size distribution is ranged between 60 and 200 nm [53, 54]. Due to their heterogeneity, separating exosomes is slightly problematic, but their isolation and enrichment are necessary to evaluate their biological functions. At present, it is not possible to isolate exosomes completely from other EVs with the current methods; thus, exosome extraction suffers from low purity, and it is important to select an appropriate isolation method for downstream analysis [44, 55]. Various isolation methods have been introduced for a variety of purposes and applications. Ultracentrifugation with at least 100,000 g is a major and common method for isolating and purifying exosomes from cell culture supernatants. Other exosome isolation methods include high performance liquid chromatography (HPLC), affinity purification with specific antibodies against CD9, CD63, CD81, and CD82, and exosome precipitation by volume excluding polymers such as polyethylene glycol (PEG). Moreover, specific exosome separation kits are commercially available which provide appropriate and efficient extraction [20, 56–58]. They are more valuable compared with ultracentrifugation because they need less time. Commercial kits are, however, more compatible with limited volumes of samples [14, 15]. After isolation, the exosomes can be identified by at least two of the following methods: scanning electron microscope (SEM), transmission electron microscope (TEM), atomic force microscope (AFM), dynamic light scattering (DLS), flow cytometry, western blot, nanoparticle tracking analysis (NTA), sequencing, qRT-PCR analysis, or enzyme-linked immunosorbent assay (ELISA) [20, 56–59]. For increasing the release of exosomes, different chemicals and environmental supplements such as gamma-irradiation, calcium ionophores, hypoxia, and acidosis conditions are required [20]. After isolation and characterization, due to instability of exosomes at room temperature and 37°C, they must be frozen before *in vivo* or *in vitro* procedures. Exosomes can be stored without cryopreservation agents for 6 months at -20°C [60]. Sokolova and coworkers [61] found that 4°C and 37°C can decrease the size of the exosomes followed by degradation or structural changes. Therefore, temperatures of less than -20°C are appropriate for exosome storage with providing stability in size and structure [20, 60].

### 2.5. Composition of the Exosomes

More than 4000 different proteins are reported in the exosomes identified by various proteomics methods such as mass spectrometry. The differences in the components of exosomes are based on different physiological/pathological conditions and certain cell types; the cell of origin imposes great impact on the exosomal contents [62, 63]. Current data from different cell types reveal that exosomes contain most of the bioactive molecules including proteins, nucleic acids, lipids, and various types of RNA including mRNAs, long noncoding RNAs (lncRNAs), microRNAs (miRNAs), transfer RNA (tRNA), mitochondrial DNA (mtDNA), cytokines, transcription factor receptors, and other bioactive substances [64, 65]. With the identification of the above compounds, the knowledge of epigenetic signaling between cells and consequent changes in biological functions is becoming more enlightened [66, 67]. Protein components of the exosomes are determined as two groups; one group is the common components that participate in the vesicle formation, secretion, and exosome biogenesis, such as programmed cell death 6 interacting protein (PDCD6IP; or ALIX) and tumor susceptibility gene 101 (TSG101) that their secretion mainly depends on several proteins like Rab GTPase proteins [9, 10], heat shock proteins (like HSP70, HSP90), tetraspanins protein superfamily (such as CD63 and CD81), and integrins [39, 68]. Cell-specific components are another group that are closely linked to antigen presenting process such as CD45 and MHC-II [39, 69–71]. Furthermore, MSC-derived microvesicles (MVs) highly express proangiogenic proteins such as basic fibroblast growth factor (bFGF), interleukin 6 (IL-6), vascular endothelial growth factor (VEGF), migration-promoting chemokines toward inflammation site such as monocyte chemokine protein-1 (MCP-1), and mitochondrial, proteasomal, and endosomal reticulum-associated proteins [72].

### 2.6. Exosomes in Tumor Progression, Angiogenesis, and Metastasis

Several studies have suggested that MSCs can help tumor progression via supporting tumor milieu, increasing tumor growth, and decreasing immune responses. In this context, MSCs are capable of migrating toward tumor sites and exert stimulatory effects on tumor growth directly by communicating with cancer cells and indirectly via secreting a number of paracrine factors, such as chemokines, cytokines, growth factors, angiogenic factors, and immune modulatory mediators [73, 74]. Nowadays, this secretome-based paracrine activity of MSCs is renowned as a cell-free strategy acting on adjacent cells or exert their effects through the blood by transferring of various molecules in exosomes [75].

Cancer progression is a dynamic and multistage process, in which exosomes play important roles. In this regard, several signaling events have been well studied, and their role in regulating the development of malignancy has been identified [76]. Growing evidence suggests that MSC-EXOs affect tumor formation, development, invasion, and drug response via transporting proteins, messenger RNA, and microRNA to recipient cells; so, understanding complex mechanisms mediated by MSC-EXOs between tumor cells and their milieu is crucial in cancer progression that can be further used to discover new approaches for cancer treatment [54, 77].

To recognize exosomes' mechanism on *in vivo* tumor growth, Zhu et al. coimplanted human gastric and colon cancer cells with MSCs or MSC-EXOs in BALB/c-nu/nu mice. Increased proliferative capacity as well as expression of important factors for tumor growth and angiogenesis including Bcl-2, phosphorylated proteins ERK1/2, CXCR4, VEGF, and MDM2 mRNA was seen in those implanting with both MSC-EXOs and tumor cells. MSC-EXOs robustly stimulated the expression of VEGF and CXCR4 via activating the ERK1/2 and p38 MAPK pathways. Accordingly, coimplanted tumor cells with MSC-exosomes have an increased tumor incidence and tumor growth *in vivo* [78]. Qi et al. found that the progression of tumor was accelerated by human bone marrow MSC-EXOs through activating signaling pathways like Hedgehog in the recipient of osteosarcoma and gastric cancer cell lines [79]. Yang et al. showed that MSC-EXO-derived-matrix metalloproteinase-2 can improve tumor growth through changing the cellular functionalities and reorganizing TME. MMP-2 and ecto-5′-nucleotidase activity can degrade collagens as structural component of basement membranes and thus alter tumor microenvironment leading to increasing tumor heterogeneity [80]. In recent years, the impact of MSC-EXOs on signal transduction has been extensively investigated. Akt, as one of the main downstream effectors of PI3K, can affect growth and cell cycle progression of tumor cells through activating multiple signal phosphorylation substrates. Gu et al. showed that induction of Akt phosphorylation by MSC-EXO leads to epithelial-to-mesenchymal transition (EMT) and gastric cancer cell regeneration [81]. MSC-EXO can transfer miRNAs, which are involved in cancer cell proliferation, differentiation, and apoptosis. Moreover, miRNAs have the ability to regulate gene expression posttranscriptionally [82]. Vallabhaneni and coworkers showed that exosomes containing miRNA-21 and -34a and tumor-supporting proteins including PDGFR-b, TIMP-1, and TIMP-2 promote the proliferation and metastasis of breast cancer cells via negative regulators of apoptosis [83].

Oncosomes (MVs that produced by cancer cells) contain carcinogenic molecules and are transferred between primary tumors and cause morphological deformation and increase anchorage-independent growth in recipient cancer cells. Tumor-derived exosomes (TD) are actively involved in inducing autocrine/paracrine oncogenesis and thus cancer progression by reprogramming stromal cells, regulating the immune system, and at the same time, enhancing angiogenesis [76] and triggering apoptosis in several tumors [59].

Cancer cells secrete higher amounts of exosomes than normal cells which indicates the significant role of exosomes in the development and progression of different types of cancers [84]. Furthermore, cancer cell-derived exosomes contain a broad range of mediators which contribute to tumor progression and metastasis [43, 85, 86]. TD exosome-derived miRNAs such as miR-9 facilitate the differentiation of fibroblasts into cancer-associated fibroblasts (CAFs) and, thus, enhance cancer development. TD-exosomes induce the differentiation of MSCs to myofibroblasts, which exhibit proangiogenic and invasive properties, and then, further promotes cancer proliferation and invasion by secreting growth factors and matrix regulatory agents [66, 87].

Several studies on cancer cells have shown that TD-exosomes can induce the proliferation of tumor cells. The proliferation and migration of human gastric cancer (GC) cells were induced through an autocrine induction when an overexpression of a long noncoding RNA named ZFAS1 in the circulating exosomes was observed [88]. TD-exosomes can affect the migration of malignant recipient cells. Exosomes created in nasopharyngeal carcinoma are transporters of signals inducing EMT. These signals include, but not limited to, hypoxia-inducible factor 1 alpha (HIF1a), matrix metalloproteinase (MMPs), Casein Kinase II, Notch1, and Annexin A2 as well as growth factors like transforming growth factor B (TGF-B), which augment the migratory capability of the tumor recipient cells [76].

Exosomes may show effects on metastatic processes such as EMT, invasion, and premetastatic niches (PMN) [89]. Exosomes derived from gastric cancer cells, BGC-823 cells, containing miR-15b-3p increases the growth of human gastric epithelium by inhibiting apoptosis and the Caspase-3/Caspase-9 signaling pathway [90]. Also, gastric cancer cell-derived exosomes transmit drug resistance such as cisplatin resistance to other susceptible clones by targeting the miR-218/HMGA1 axis in sensitive cells (MGC803 cell) [91]. PMN, which has distinct characteristics from the natural tissue environment such as immunosuppressive, angiogenic, and organotropism properties, is also influenced by TD exosomes. Exosomes in PMN not only support stromal components through stromal regeneration by CAF, MSC, and ECM balance and angiogenesis but also suppress immune system through a variety of mechanisms including polarization toward tumor-associated macrophage (TAM) and tumor-associated neutrophil (TAN), inhibiting immune cells such as DC and T lymphocytes maturation, and inducing myeloid derived suppressor cells (MDSCs) [89]. Gastric cancer cells' exosomes activate macrophages which cause significant increase in the expression of proinflammatory factors such as NF-*κ*B leading to tumor cells proliferation and migration [92].

In a study on pancreatic cancer, exosomes derived from cancer cells facilitate the metastasis of tumor by inducing the generation of tumor-associated cells such as CAFs, TAMs, and cancer initiating cells (CICs) that may strengthen the invasion growth, proliferation, resistance to drugs, and consequently, EMT and metastasis. TAMs are a group of macrophages that penetrate TME and cause resistance to chemotherapy, angiogenesis, and migration. TAM-derived exosomes contain miR-501-3p which inhibits the expression of TGFBR3, activates TGF-*β* signaling, and causes the metastasis of pancreatic cancer xenografts in nude mice [93].

Exosomes may play pivotal roles as a bridge between cancer cells and various immune cells such as macrophages, neutrophils, natural killer cells (NK), dendritic cells, and T cells. In the context of epithelial ovarian cancer, macrophages are attracted toward tumor by gaining miR-222-3p from exosomes and differentiate toward M2 macrophages in a SOCS3/STAT3 signal-dependent pathway. M2 macrophages with immunosuppressive phenotype, CD206^high^Arg-1^high^IL-10^high^, induce angiogenesis and lymphangiogenesis in the microenvironment and promote the progression of ovarian cancer [66, 94]. TD-exosomes attenuate immune responses and then facilitate tumorigenesis by stopping differentiation of monocyte into DCs, subsequently suppressing T cell activity, proliferation, and anticancer cytolytic functions. Production of inhibitory cytokines such as PGE2 and TGF-*β* besides low expression of costimulatory molecules is the properties of DCs generated in the presence of TD exosomes [95].

One of the essential multistep physiological processes in tumorigenesis is angiogenesis. Exosomes have several angiogenic factors including VEGF, IL-8, TGF-*β*, and fibroblast growth factor (FGF), which enhance proliferation and migration of endothelial cells and are necessary to induce tumor angiogenesis [22, 59].

Exosomes released by cancer cells also enhance tumor growth and aggressive behavior by altering different types of stromal cells and activating endothelial cells through autocrine VEGF signaling to increase tumor angiogenesis [96, 97]. MSC-EXOs motivate angiogenesis by increasing the production of VEGF in tumor cells and stimulating mitogen-activated protein kinase pathways with ERK1/2 and P38. In one study, platelet-derived growth factor (PDGF) originating from adipose MSC-EXOs, which are rich in proangiogenic factors, causes the development of angiogenesis [98]. Injection of MSC-EXOs into a mouse stroke model showed angiogenesis, regeneration, and neurogenesis stimulation, and consequently, attenuation of symptoms. Also, MSCs boost proliferation of endothelial cells and capillary network formation by producing exosomes that transmit miRNAs to target cells [14]. According to bioinformatics analysis, Ferguson et al. suggested that some of MSC-EXOs induce angiogenesis by targeting various genes including Wnt signaling, profibrotic signaling via TGF-*β*, and PDGF related to angiogenesis and vascular formation. Other factors including carcinogenic proteins, cytokines, and adhesion molecules can be involved in exosome-mediated angiogenesis as well [99]. TD-exosomes containing miR-17-92 cluster can induce endothelial migration and tube formation due to increased expression of vascular cell adhesion molecule-1 (VCAM-1) and intercellular adhesion molecule-1 (ICAM-1) [100].

The presence of a favorable niche as special microenvironment is necessary for survival, proliferation, and metastasis of tumor cells. Numerous studies have shown the role of MSC-EXOs in invasion and site formation before metastasis. For instance, MCF7 breast cancer cell line showed enhanced migration capacity after exposure to MSC-EXOs [54]. MSC-EXO facilitates the growth and migration of breast tumor cells by activating the Wnt signaling pathway [14, 101]. Also, it has been clarified that MSC-EXOs deliver miR-221 to human gastric cancer HGC-27 cells inducing tumor cell growth and migration [102].

Drug resistance is a major challenge for cancer therapy as well. Several studies reveal that exosomes are involved in the modulation of chemosensitivity by transferring the resistant phenotype to recipient cells. Transport of ncRNAs (noncoding RNAs), including miRNAs and lncRNAs (long noncoding RNAs), mediated by exosomes, is believed to be an effective mechanism for acquiring drug resistance in cancer cells [103]. In ovarian cancer, exosomal transfer of miR-433 can promote paclitaxel resistance through the induction of cell senescence related genes including cyclin-dependent kinase 6 (CDK6), MAPK14, E2F3, and CDKN2A. So, the induction of cellular senescence and subsequent altered cell signaling has been shown to correlate with changes in the epigenome of cells and to promote further cancer progression [104].

Exosomal lncRNA-SNHG14 (lncRNA-small nucleolar RNA host gene 14) in breast cancer promotes trastuzumab resistance in HER2+ patients by targeting the apoptosis regulator Bcl-2 (Bcl-2)/apoptosis regulator BAX (Bax) signaling pathway. Furthermore, extracellular lncRNA-SNHG14 was able to be incorporated into exosomes and transmitted to sensitive cells, thus spreading trastuzumab resistance [105, 106]. Zhang et al. indicated the role of exosomal lnc SBF2-AS1 (long noncoding RNA SBF2 antisense RNA 1) in temozolomide (TMZ) resistance of glioblastoma (GBM) cells. Transcription factor zinc finger E-box binding homeobox 1 (ZEB1) directly binds to the promoter of SBF2-AS1 regulating its expression level and resulting in TMZ resistance in GBM cells [107].

Transferring multidrug resistance- (MDR-) associated proteins such as P-glycoprotein (P-gp), a glycoprotein encoded by ABCB1 gene, by TD exosomes to target cells is another mechanism in chemotherapeutic resistance in tumor cells. Indeed, these proteins cause drug efflux and confer resistance by preventing sufficient accumulation of anticancer drugs within the cells [108].  Figure 2 represents an overview of exosome functions in TME.

### 2.7. Antitumor Effects of Exosomes

As exosomes contain biologically active molecules can act as therapeutic tools for exogenous drugs and stabilize the drug in vivo. By changing the traditional mode of drug delivery to targeted therapy, exosomes become important tools to promote the development of personalized medicine. As the biological effects of exosomes have been discovered, the functional roles of these small secretory vesicles with miscellaneous contents in human health and cancer have been increasingly investigated [23].

Exosomes as medicinal cell-free products are in fact the main means of paracrine effect of MSCs that involve in cell-cell interactions [20, 109], and many therapeutic effects of MSCs mostly attribute to the MSC-EXOs [110, 111]. The use of MSC-derived secretome in therapy offers several advantages compared with MSCs including the suppression of apoptosis, stimulation of remodeling of the extracellular matrix, and angiogenesis [112, 113]. Therefore, it is generally safer than using cells owing to the lack of self-replicability and tumor formation and low emboli formation [113]. Although MSC-EXOs show tumor-boosting effects in various types of cancers, there is also evidence for antitumor activity of MSC-EXO. Wu and colleagues [114] reported that the growth of bladder carcinoma cells was inhibited by EVs derived from human umbilical cord Wharton's jelly MSCs mediating by downregulation of phosphorylation of Akt kinase protein and the upregulation of cleaved caspase-3. Likewise, miR-145 in exosomes from adipose-MSC inhibits prostate cancer via reducing the activation of Bcl-xL and promoting apoptosis through the caspase-3/7 pathway [115]. Also, EVs extracted from normal human BM-MSCs hinder the proliferation, but promote the apoptosis of different tumor cells in some tissues such as liver and ovary and Kaposi's sarcoma cell lines [116]. The role of MSC-EXO in angiogenesis and neovascularization is still controversial [54]. Lee et al. showed that MSC-EXO inhibits vascular formation by delivering miR-16 and regulating VEGF in the tumor microenvironment [117]. In parallel, Huang et al. showed that MSC-EXO can inhibit hypoxia-induced mitogenic factor (HIMF) and Smad2 resulting in antivascular regeneration [118]. The status of donor seems to be important for the tumor-suppressive or tumor-promoting effects. Roccaro and coworkers observed that EVs from BM-MSCs in patients with multiple myeloma support the tumor progression, whereas EVs isolated from normal individuals inhibited the development of tumor by lowering the miR-15a transfer [119]. Multiple studies on exosomes revealed the dual role for exosomes in promoting or suppressing cancer depending on the type and stage of cancer and the source of exosome [96, 120].

## 3. Conclusion

As intriguing biological nanocargoes, exosomes have recently received extensive scientific attention. They play crucial roles in cell phenotype and controlling various vital biological processes as they are tools for cell-to-cell communication. Regarding the content, exosomes are capable of stimulating cancer progression and metastasis through induction of EMT, invasion, angiogenesis, immune modulation, and even drug resistance. Cancer cells and MSC-EXOs promote the development and metastasis of cancer by suppressing the immune responses and enhancing resistance to chemotherapy through eliminating chemical anticancer drugs. On the other hand, there is also evidence for antitumor activity of MSC-EXOs in some types of tumors such as prostate and bladder cancers. The source of MSCs or the condition of the donor seems to be perceived as a determinative factor for tumor suppressive or progressive role of MSC-EXOs. Considering the antitumor effects of exosomes and their capability of easily reaching the bulk of solid tumors, they can be engineered as potential drug delivery vehicles or cell free vaccines providing alternative strategies for exosome-based anticancer therapies. Routine cell-based therapies could be merely replaced by exosome therapy and MSC-EXOs provide scientists with fascinating information on the content and mechanism of action of exosomes. However, due to the dual role of exosomes, more detailed studies on these mysterious bullets are undoubtedly needed. Accordingly, optimizing the methods to improve the yield and purity of exosomes would be the most important priority both for seeking the mechanism of action and for therapeutic purposes.

## Figures and Tables

**Figure 1:** Exosome biogenesis and secretion. First, insertion of the cell membrane leads to the formation of early endosomes, and then, endosomes containing RNA and cytosolic proteins are transformed into MVB structures with dynamic subcellular structures. After that, MVBs can be fused with lysosomes and degraded or secreted by plasma membranes and formed exosomes. Finally, exosomes release their cargo, such as DNA, microRNA, and proteins, into the recipient cell in a variety of ways. MVBs: multivesicular bodies.

**Figure 2:** An overview of exosome functions. MSC-EXOs and tumor-derived exosomes exert various effects on recipient cell through different target/pathway. The interaction between exosome and other cells of TME may result in proliferation, tumor growth, metastasis, and drug resistance. Arrow in the figure above: stimulator. MSC-EXOs: MSC's exosomes; TME: tumor microenvironment; VEGF: vascular endothelial growth factor; CXCR4: C-X-C chemokine receptor type 4; ERK1/2: extracellular signal-regulated kinases 1/2; MAPK: mitogen-activated protein kinases; AKT: protein kinase B; EMT: epithelial–mesenchymal transition; mir: microRNA; MDR: multidrug resistance protein.

**Table 1:** Features of extracellular vesicle subtypes.

	Exosomes	Microvesicles	Apoptotic bodies
Mechanism of formation	Fusion of MVBs with the plasma membrane	Outward blebbing of the plasma membrane	Product of programmed cell death and cell shrinkage
Intracellular origin	Endosomes	Plasma membranes	Plasma membrane, cellular fragments
Size	40–150 nm	150–1000 nm	100–2000 nm
Density	1.13–1.19 g/ml	1.04–1.07 g/ml	1.16–1.28 g/ml
Shape	Spheroid or “cup-shaped”	Irregular	Variable, heterogeneous
Composition	Proteins, nucleic acids, lipids and metabolites, various types of RNA including mRNAs, miRNAs and tRNA, mtDNA, cytokines, transcription factor receptors	Proteins, nucleic acids, lipids and metabolites, cytoplasmic material	DNA fragments and histone, chromatin remnants, cytosol portions, degraded proteins
Typical markers	Tetraspanins (CD63, CD81, CD82, and CD9), ESCRT proteins (ESCRT-3, Alix, TSG101), heat shock proteins (Hsp60, Hsp70, and Hsp90)	Integrins, selectins, CD40 ligand, Flotillin-2, ADP-ribosylation factor 6 (ARF6), bFGF, IL-6, VEGF, MMPs	Annexin V, phosphatidylserine histones
Function	Cell–cell communication, regulate intercellular signal transduction, cancer cell-induced angiogenesis, promotion of cancer cell growth	Cell–cell communication, cancer cell-induced angiogenesis, promotion of cancer cell growth	Facilitate clearance of apoptotic cells, maintaining regular cell populations in tissues for homeostatic mechanism, intercellular communication for immune regulation
Isolation method	Immunoprecipitation (ExoQuick1), ultracentrifugation (>100,000 g)	Immunoaffinity chromatography ultracentrifugation (10,000-100,000 g)	No standardized protocol, sometimes ultracentrifugation (1,200-100,000 g)
Detection technology	Electron microscopy and western blotting (with specific exosome markers), TEM, SEM, flow cytometry, ELISA	Electron microscopy, TEM, SEM, flow cytometry for microvesicles >300 nm	Electron microscopy, flow cytometry and fluorescence microscopy
References	[16, 21–28]	[4, 24, 26–30]	[16, 24, 26–28, 31, 32]

## Abbreviations

MSCs: Mesenchymal stem cells
MSC-EXO: Exosome-derived mesenchymal stem cells
TME: Tumor microenvironment
EVs: Extracellular vesicles
ISEV: International Society for Extracellular Vesicles
MVBs: Multicellular bodies
sEV: Small extracellular vesicles
DCs: Dendritic cells
NK: Natural killer
APCs: Antigen-presenting cells
ESEs: Early sorting endosomes
LSEs: Late sorting endosomes
ESCRT: Endosomal sorting complexes required for transport dependent
HPLC: High-performance liquid chromatography
PEG: Polyethylene glycol
SEM: Scanning electron microscope
TEM: Transmission electron microscope
AFM: Atomic force microscope
DLS: Dynamic light scattering
NTA: Nanoparticle tracking analysis sequencing
ELISA: Enzyme-linked immunosorbent assay
lncRNAs: Long noncoding RNAs
miRNAs: MicroRNAs
tRNA: Transfer RNA
mtDNA: Mitochondrial DNA
PDCD6IP: Programmed cell death 6 interacting protein
TSG101: Tumor susceptibility gene 101
HSP: Heat shock proteins
FGF: Fibroblast growth factor
PDGF: Platelet-derived growth factor
VEGF: Vascular endothelial growth factor
MCP-1: Monocyte chemokine protein-1
EMT: Epithelial-to-mesenchymal transmission
TD: Tumor-derived exosomes
CAFs: Cancer-associated fibroblasts
GC: Gastric cancer
HIF1a: Hypoxia-inducible factor 1 alpha
MMPs: Matrix metalloproteinase
TGF-b: Transforming growth factor B
PMN: Premetastatic niches
TAM: Toward tumor-associated macrophage
TAN: Tumor-associated neutrophil
MDSCs: Myeloid-derived suppressor cells
CICs: Cancer initiating cells
VCAM-1: Vascular cell adhesion molecule-1
ICAM-1: Intercellular adhesion molecule-1.
